# Investigating the EKC hypothesis with renewable energy, nuclear energy, and R&D for EU: fresh panel evidence

**DOI:** 10.1016/j.heliyon.2022.e12447

**Published:** 2022-12-22

**Authors:** Liton Chandra Voumik, Mahbubur Rahman, Salma Akter

**Affiliations:** Department of Economics, Noakhali Science and Technology University, Bangladesh

**Keywords:** CS-ARDL approach, CO_2_ emissions, Environmental degradation, EKC, Nuclear energy, Renewable energy consumption

## Abstract

The European Union (EU) is extremely concerned about the environmental harm caused by rising CO_2_ emissions and other factors. The EU has to uncover factors that decrease pollution before it's too late to achieve long-term sustainable growth. The paper applies the environmental Kuznets curve (EKC) hypothesis to examine the dynamic connection between GDP, energy use, energy intensity, research and development (R&D), and CO_2_ emissions. Data from 34 countries in the EU, spanning from 1990 to 2021, were applied. EU countries are very interdependent on one another due to tourism, trade, education, religion, and culture. Therefore, tests for cross-sectional dependency (CSD) and slope heterogeneity (SH) are used in this research. After establishing the presence of CSD and SH issues, the study employed second-generation unit root and cointegration tests. In response to these concerns, the study implemented a novel cross-section autoregressive distributed-lag model (CS-ARDL) method. There exists a U-shaped quadratic link between environmental pollution and wealth. That rules out the existence of the EKC hypothesis in the EU. This means that when income grows, pollution will drop up to a certain point, and then it will begin to climb again. Long-term pollution is reduced by the use of renewable energy and R&D. On the other hand, energy intensity increases CO_2_ emissions. The article also applied the CCEMG, AMG, and MG estimators to test the robustness. The CS-ARDL methodology demonstrates that increasing national income, nuclear energy, and investment in R&D alone will not be sufficient to fulfill environmental needs and that the use of alternative renewable energy sources is the greatest approach to mitigate environmental deterioration in the EU. The AMG, MG, and CCEMG estimators all agree that switching to renewable energy is the most effective strategy to lower emissions. This research offers crucial guidelines for advancing environmental policy and realizing sustainable development. Discussion, policy recommendations, and future research based on the findings are presented.

## 1 Introduction

For the last few months, European nations have been facing a tragic war between the Russian Federation and Ukraine. Both nations are the main suppliers of energy for the EU nations. That's why they are not able to receive energy from this two-war-engaged country. So, searching for *renewable energy* can be a new pathway for EU countries. This pathway can be helpful to alleviate the emission of greenhouse gases, which are harmful to the ozone layer and also responsible for an increase in the earth's temperature. An economy aims to achieve the desired level of economic development and growth and to keep that level constant. Although economic development benefits society, it has negative environmental consequences. The relationship between these processes and the deterioration of the environment is still up for debate among academics and politicians. Environmental pollution and damage to the environment are two of the most crucial of these. The whole globe's energy needs are largely fulfilled by fossil fuels, whose supply is quickly depleting. Environmental issues, including rising CO_2_ *emissions* and the effects of greenhouse gases, are also major concerns for the world. The EU will emit approximately 2.73 billion metric tons of CO_2_ in 2021. This was six times more than the emission of carbon dioxide in 2020 by the EU. In 2021, the European Union consumed 6.62 Exajoules of *nuclear energy (**IEA, 2022**)*. Economic theory suggests that an increase in the use of any product increases its cost. Therefore, the overuse of non-renewable energy sources, like natural gas, coal, oil, and other fossil fuels, is expected to cause an increase in energy costs over time. The gas emissions from these sources raise the level of carbon dioxide, which damages the environment and increases the demand for energy for economic activity. According to several empirical studies, the environment primarily hampers economic development to a particular level but then improves.

The Kuznets curve was developed by Kuznets (1955 and 1963), who also reported that the EKC hypothesis is a postulated link between several measures of environmental deterioration and per capita income. While early economic growth is accompanied by a rise in pollution emissions and a loss in environmental quality, later stages of development are associated with an improvement in both. That's why the EKC is an inverted U-shaped curve. The EKC hypothesis is famous for explaining the relation between two important indicators, which are income and pollution. In recent years, this relationship has mostly concerned researchers as well as policymakers. Grossman and Krueger (1991) narrated and proved that environmental qualities are thought to decline in the initial stages of economic growth in a country, then reach their peak, and after that, environmental quality improves with the improvement of the economic condition of that country, and an inverted U-shaped curve is applied to symbolize it. Chien et al. (2021) explained a famous theory that states that the EKC hypothesis posits a link between environmental deterioration and economic expansion. The reviewed studies on energy and the environment support the viability of the EKC theory. The availability of *renewable energy* will be created by providing subsidies, tax holidays, and other more effective policies and guidelines to attract investment in the renewable energy sector, which will play an alternative role as a source of conventional energy in European Union countries (Paramati et al., 2021). Destek and Sinha (2020) developed an ecological footprint that can be more accurately representative of the environment. It is examined how real income, real income squared, consumption of refillable energy, usage of non-refillable energy, ecological footprint, and trade openness, relate to one another using the analysis of cross-sectional dependency taken into consideration by second-generation panel data methods. The overconsumption of *renewable energy*, as well as trade openness, decreases the ecological footprint, whereas environmental pollution increases with the overuse of *non-renewable energy*.

As a result, a fresh look at the interplay of renewables, GDP growth, nonrenewables use, nuclear power, innovation, and carbon dioxide emissions are urgently required. In the framework of the EU, our research aims to provide light on the connection between CO_2_ emissions and alternative energy sources, GDP growth, nonrenewable energy use, nuclear power, and technological advancement. In this analysis, we test the robustness of the EKC hypothesis using several fresh estimators for the EU member states. Though the EU is considered an environmentally conscious region, its massive GDP, increasing consumption of renewable, non-renewable, and nuclear energy, and spending on R&D can impact the environment. At present, energy is the biggest concern for the environment in Europe. European countries have comprehensive environmental laws, but it is important to find out which factors are responsible for environmental degradation so that countries can take initiatives to protect the environment. For these reasons, this paper prefers to describe the CO2 emissions of European countries that are favored to generate efficient policy recommendations. Furthermore, this study included renewable energy, energy intensity, nuclear energy, and R&D as control variables to track their effects on the state of the ecosystem. This research could help European policymakers reduce environmental degradation, choose energy policies, and implement sustainable growth. The CSD and SH tests were used in the study because EU countries are highly interconnected through tourism, trade, education, religion, and culture. Most of the previous tests did not consider these problems. Also, this paper considers the second-generation unit root and the cointegration test. Concerning all of these problems, the research applied the CS-ARDL, AMG, MG, and CCEMG estimators.

The research gap and the EKC literature designed for European nations are summarized in Section 2. Later, Section 3 introduces sources of data and theoretical, and empirical frameworks. Tests and empirical findings are presented in Section 4. A discussion of the findings is described in Section 5. In the end, this paper is accomplished with the conclusion and policy implications in Sections 6 and 7. Research limitations and future research are also included.

## 2 Literature review

Prior studies with variables eventually argued and provided knowledge of the EKC hypothesis. Many European nations have set goals to spread *renewable energy* because of its key role in alleviating carbon dioxide emissions. Bezi (2022) stated that technological innovation was effective in reducing carbon emissions in the EU from 2012 to 2019 using the panel GMM method and that EU nations should increase innovative activity to achieve a sustainable environment. Ozgur et al. (2022) used the Fourier ARDL method to examine how nuclear power affected CO_2_ emissions in India between 1970 and 2016, concluding that nuclear energy and GDP2 were beneficial in reducing CO_2_, but GDP increases environmental deterioration. Voumik and Sultana (2022) applied a CS-ARDL model to examine the relationship between urbanization, *renewable energy*, electrification, industrialization, and environmental degradation in the BRICS countries from 1972 to 2021. They found that while other variables in the BRICS countries stimulate environmental degradation, *renewable energy* significantly slows it down. An analysis utilizing the ARDL approach looks at how population, energy use, and economic development in Bah have an impact on CO_2_ *emissions* throughout the period from 1971 to 2020 (Voumik et al., 2022a). The research's findings demonstrated that over time, the population has little effect on carbon emissions, while fossil fuels have a negative influence on the environment. In addition, a variety of development strategies support income and reduce carbon emissions.

Zeqiraj et al. (2020) applied the familiar (CS-ARDL) for 23 EU nations from 1980–2016 to analyze the outcome of innovation in technology, the stock market, and sustainable energy on the predominance of carbon dioxide. They found that the stock market increases the volume of carbon dioxide in the air. Though carbon dioxide emissions can be reduced through the use of renewable energy, in addition, better environmental and energy policies should be recommended to ensure the prolongation of the stock market, which will ensure the reduction of carbon emissions. Su et al. (2020) examined how energy efficacy and the usage of renewable resources contribute to mitigating the emission of GHGs. Between 2005 and 2016, the European Union experienced a series of successes. Their findings revealed that GHG reductions can only be achieved by increasing the share of renewable energy in ultimate energy consumption and by reducing power consumption. Paramati et al. (2021) analyzed how environmental sustainability is impacted by *research and development*. Their findings show the more money spent on R&D, the more renewable energy is used, which significantly reduces GHGs in European countries from 1998 to 2014. Aydin et al. (2019) tested EKC for EF. They used data from 1990 to 2013 for a panel data analysis of 26 EU nations. In detail, six sub-elements of EF were differently studied, and the results suggested that there exists an invalid EKC, which is obvious with the model of PSTR. In the meantime, a widespread panel data analysis of 131 countries from 1971 to 2017 decomposed the exordiums of economic development to determine EF by using the FEM, REM, POLSM, and GMM models. Majeed and Mazhar (2019) found that financial improvement is encouraging for decreasing global EF, even if economic development and energy use raise it. In BRICS countries, Dogan et al. (2020) used energy structure and energy intensity to re-inquire EKC, where EKC was discerned to be voided from 1980 to 2014 using the AMG, DOLS, and FMOLS models. Furthermore, a study of the BRICS economies found that energy use, urbanization, and natural resource rents are determinants of EF. Awais and Wang (2019) also evaluated the importance of government subsidies to reduce CO_2_ *emissions* from 1996–2017. According to their report, when governance quality is better, this helps to reduce CO_2_ emissions in BRICS nations, which in turn helps to decrease environmental degradation in BRICS nations. By applying the AMG estimation, Akif and Asumadu (2019) tested the nature of energy, growth, and financial progress in the panel data investigation of ecological footprint. From 1977 to 2013, EKC in the shape of an inverted U is evident in recently industrialized nations. From 1984 to 2015 in the United States (US), Bildirici (2017) examined the connection between the consumption of biofuels, militarization, CO_2_ *emissions*, and growth of the economy by applying the ARDL, CCR, DOLS, FMOLS, and MWALD F tests developed by Toda Yamamoto and Rao. It revealed that there is a causal association between CO_2_ *emissions* and militarization. In policy recommendations, it was stated that if it is possible to reduce defense expenditures, then CO_2_ *emissions* can be reduced or the usage of bio-fuel energy can be expanded.

Abbasi et al. (2020) anatomized the data for eight ASEAN economies from 1982–2017. The Granger Causality Test and Panel Co-integration Test revealed that energy use had a significant impact on CO2 in the eight ASEAN nations. Liu et al. (2020) studied the connection between *CO2 emissions* and globalization from 1970 to 2015, taking into account the G-7 countries. The author's results suggest that urbanization initially increased *CO2* levels but ultimately led to a reduction in *CO2 emissions* after they reached a certain level. Anser et al. (2019) used unobserved panel heterogeneity to support the accuracy of the EKC across the board for the G-7 nations. Ari and Şentürk (2020) used a variety of group structural breaks and lengthy estimators, but they were unable to corroborate the EKC for any of the G-7 nations. Nyla Saleem and Shujah-ur-Rahman (2019) observed how the BRICS nations' bio- and human capacities impact the environment utilizing the first-generation co-integration tests. Estimates led to the discovery of the EKC, a backward U-shaped curve. The most recent index, created by Sun et al. (2020), which measures human resources based on the number of patents for every million comprehensive *RD* employees, educated the public with the creative notion of human capital. With the use of the model's human capital, the study's findings indicated EKC survival. Wang et al. (2020) tested the EKC hypothesis, including all seven nations, using a dynamic random regression approach. Zaidi et al. (2019) investigated the global integration emissions nexus for APEC nations from 1990 to 2016. The authors discovered that urbanization reduced emissions of *CO2*. Moreover, the results of this research validated the EKC model. Shahbaz et al. (2019) used the modified technique of consequences method to demonstrate the EKC for all the countries in the G7 group. Sehid (2021) employed the startup panel rolling screen test of causality for these nations, and only the United States and Japan validated this theory. Bhatti et al. (2020) also looked at the ASEAN nations, and based on the results of panel ARDL estimation using panel data, the authors determined that globalization was responsible for reducing carbon emissions in the ASEAN nations analyzed.

Amarante et al. (2021) illustrated that economic extension and CO_2_ are linked in both directions. The amount of *nonrenewable energy* used also influences CO_2_ *emissions* and economic growth favorably. However, using *renewable energy* hurts CO_2_ *emissions* while having a favorable impact on economic growth. Additionally, economic expansion promotes the use of both renewable and nonrenewable energies. Safi et al. (2021) narrated that environmental taxes, environmental *RD*, and exports greatly lowered carbon emissions in the short- and long-term, whereas *GDP* and imports significantly increased carbon emissions in G-7 countries from 1990 to 2019. Tao et al. (2021) analyzed the CS-ARDL method for G-7 countries and narrated how eco-innovations and environmental taxes significantly help to alleviate CO_2_ *emissions*. Khan et al. (2019) conducted dynamic ARDL simulations to analyze data for South Asian countries like Pakistan from 1971 to 2016 to predict the association between foreign direct investment, globalization, energy use, globalization, *FDI*, and CO_2_ *emissions*. The researchers noted that all of the variables stated above had a favorable contribution to CO_2_ *emissions* in Pakistan. Amour et al. (2019) tested the EKC for a Eurasian country like Turkey from 1980 to 2014 by including borrowing costs and energy usage statistics. Their study supported the EKC in 30 out of 50 states in the United States by using an estimator of the augmented mean group, while the CCEMG approach was applied to maintain the EKC in 10 states (Atasoy, 2017). Zhang et al. (2019) applied the ARDL test to study the case of China. This result also confirmed the EKC's existence. But a study conducted by Chen et al. (2019) revealed that the EKC was invalid for the world's most populous country, China, from the years 1980 to 2014 in the model along with economic growth and traditional use of energy, while the addition of the long-term viability of the EKC was also supported by sustainable energy in the model. In addition, the independent factors that were considered and selected for this analysis were those that emerged from the assessment of the remaining literature as having the most significant effects on carbon dioxide emissions. This study can be traced by the next research, and in this way, the narrowness of this valuable investigation could have been seen.

Through the literature review, the environmental impact of ${\mathrm{CO}}_{2}$ *emissions* in various countries and how they can be mitigated are discussed. But there is a little gap here. A few papers have addressed how ${\mathrm{CO}}_{2}$ *emissions* can be reduced by green technologies, and a few researchers have investigated the European Union. Therefore, this paper has tried to fill the gap and shows how *renewable energy, economic growth, nuclear energy, and R&D* impact ${\mathrm{CO}}_{2}$ *emissions* through the CS-ARDL model; very little work has been done on the European Union, and it also tries to show the rationality of the EKC theory.

## 3 Methodology

### 3.1 Data

The World Development Indicator was used as the main source for all of the variables. The particulars of the variables, in addition to certain descriptive statistics, have been laid out in Table 1, Table 2 to make things easier for our readers. The yearly data were collected from 34 European countries, and the period is from 1990 to 2021.

**Table 1:** Variables' names and particulars.

Variables	Short form	Indicators
CO_2_*emission*	*L*CO_2_	CO_2_*emission* (kt)
*GDP*	*LGDP*	*GDP* (constant 2015 US$)
*GDP square*	*LGDP*^2^	Trade (% of *GDP*)
*Renewable energy*	*LREN*	Percentage of the total energy used that comes from renewable sources.
*Energy intensity*	*LENER*	Primary energy intensity level (MJ/$2017 PPP GDP)
*Nuclear energy*	*LNUC*	Nuclear and alternative energy (% of total energy use)
*Research and Development*	*LR&D*	Research and Development

**Table 2:** Descriptive statistics.

Variables	N	mean	SD	min	max
*L*CO_2_	957	11.11	1.926	4.942	14.59
*LGDP*	1,002	26.02	1.803	21.02	28.91
LGDP^2^	1,002	680.1	91.66	441.7	835.9
*LREN*	961	2.131	1.644	−5.021	4.359
*LENER*	824	1.114	0.536	2.461	0.808
*LNUC*	788	1.784	1.780	−10.12	3.924
*LR&D*	684	0.154	0.745	−3.163	1.510
*Number of Countries*	34				

Table 1 contains the variable lists that were utilized for this study, as well as the log of the short form. Table 2 contains an overview of the statistical information about all of the variables. In the summary data, the log of GDP_2_ has the greatest values, while the log of R&D has the lowest values. In contrast to the other standard variables, which can only fall within the range of 0.536 to 1.926 in terms of standard deviation, GDP squared is considered too high. The highest number of observations for GDP is 1002, while the lowest number of observations is 684 for R&D. This is panel data that is not balanced.

### 3.2 Theoretical outline and EKC hypothesis

The EKC proposition states that the environment initially causes more corrosion as an economy grows, but pollution levels gradually decline as income levels rise. EKC makes an important connection between environmental deterioration and income growth. The EKC proposition mainly discusses the relationship between income and environmental degradation. It is assumed that ecological pressure increases with the economic development of a country and then decreases with the further economic development of that country. EKC represents the reversed U-shaped curve. In this study, the research aims to explain the EU nation's influence on the reduction of *CO2* on the environment, mainly on the earth's air, water, and soil. It is not possible to save the environment if rich countries such as the EU use nonrenewable energy. If advanced countries rise renewable energy use in all sectors of production and consumption, the goal of sustainable development may be achievable. The per capita income in European countries is high. If EKC exists in EU countries, income can be a good indicator to minimize pollution. Furthermore, income cannot be the only indicator used to combat pollution in Europe; there are other important variables to consider. So, the research considers renewable energy, energy intensity, R&D, and nuclear energy variables to measure the dynamic linkage with CO_2_ emissions. When it comes to the EKC, according to Grossman and Krueger (1991), the association between environmental deterioration and per capita income has an “inverted U” shape. The next step is to incorporate our relevant independent variables and CO_2_ emissions into an equation.

To represent the aforementioned analysis, the following equation (1) is formed:

(1) Environmental degradation=f(GDP,GDP2,REN,ENER,NUC,RD)

We can rewrite the aforementioned equation in the EKC format in Eq. (2):

(2) $$ED_{i,t}=\beta_{0}+\beta_{1}{\mathrm{GDP}}_{i,t}+\beta_{2}{\mathrm{GDP2}}_{i,t}+\beta_{3}Z_{it}+\varepsilon_{it}$$

where *ED* means environmental degradation. *GDP* and *GDP2* explain income level and its square, respectively. Z includes other variables that impact environmental pollution, such as *renewable energy, nuclear and alternative energy, energy intensity, R&D*, etc.

The following Equation (3) is the details form of Equation (2)

(3) $${\mathrm{CO}}_{2i,t}=\beta_{0}+\beta_{1}{\mathrm{GDP}}_{it}+\beta_{2}{\mathrm{GDP}}_{it}^{2}+\beta_{3}{\mathrm{REN}}_{it}+\beta_{4}{\mathrm{ENER}}_{it}+\beta_{5}{\mathrm{NUC}}_{it}\;\;+\beta_{5}{\mathrm{RD}}_{it}+E_{it}$$

Here, ${\mathrm{CO}}_{2}=\text{Carbon emission}$, REN=Renewable energy, GDP=GrossDomestic Product, ENER=Energy intensity, and NUC=Nuclear energy.

The long form of equation (4) is constructed as follows to assess if the EKC hypothesis is:

(4) $$\text{L}{\mathrm{CO}}_{2i,t}=\beta_{0}+\beta_{1}L\mathrm{GDPit}+\beta_{2}L{\mathrm{GDP}}_{it}^{2}+\beta_{3}L{\mathrm{REN}}_{it}+\beta_{4}L{\mathrm{ENER}}_{it}\;\;+\beta_{5}L{\mathrm{NUC}}_{it}+\beta_{6}L{\mathrm{RD}}_{it}+E_{it}$$

Here $\beta_{0}$ is the intercept term.

In this research, $\beta_{1}$ *to* $\beta_{6}$ are slope coefficients. Here, *i* and *t* characterize the cross sections and time indicators.

### 3.3 Econometric methodology

Panel configurations were used to generate the study's data. In this study, pretests were utilized to validate the data to ensure its accuracy. Though almost all of the EU countries are developed, their economies, energy consumption, and other attributes are not similar. So, the slope heterogeneity test is important here. Second, EU countries are highly interconnected with tourism, trade, education, and other factors. As a result, CSD testing is critical in this case. In the third phase, we will confirm the consistency of the data. The panel cointegration test is going to be employed for the fourth step of the process. In the final step of this research, an econometric model will be chosen to analyze the long-term causal relationships between the dependent variable and the independent variables. This decision will be based on the results of the tests that came before it. To do this, the research used tests of the second generation. Estimators for the AMG, MG, and CCEMG were utilized in the study, which was conducted using the CS-ARDL approach. To validate the findings of the study, the most recent three tests are analyzed. The methodology's flow chart is depicted in Fig. 1, below.

**Figure 1:** Steps of methodology.

#### 3.3.1 Slope homogeneity test

When working with panel data, taking into account the slope heterogeneity of the data is a significant concern. Following that, the Pesaran and Yamagata (2008) analysis for slope homogeneity is carried out. When computing the outcomes of this test, the weighted slope of each participant is taken into consideration. Following Equation (5) shows the slope heterogeneity:

(5) $$\overset{ˇ}{\Delta }=\sqrt{N}(\frac{N^{-1}S\text{\%}-k}{\sqrt{2k}})\;\text{and}\;{\overset{ˇ}{\Delta }}_{\mathrm{adj}}=\sqrt{N}(\frac{N^{-1}S\text{\%}-k}{\sqrt{\frac{2k(T-k-1)}{T+1}}})$$

#### 3.3.2 CSD test

It is expected that there will be a rise in the amount of cross-sectional dependency in panel data if there is an increase in the level of economic integration and the elimination of other obstacles (Tufail et al., 2021). If we choose to ignore the issue and pretend that each cross-section exists independently of the others, then CSD can lead to information that is biased, deceptive, and inconsistent (Westerlund and Edgerton, 2008). This work uses large panel data econometrics with CSD of weakly exogenous variables to analyze CSD (Pesaran, 2015). Before using the panel data econometric second-generation unit root tests, it is necessary to first ensure that slope homogeneity and cross-sectional dependence are present in the data. For CSD tests, Equation (6) shows the method:

(6) $$\mathrm{CSD}=\sqrt{\frac{2T}{N(N-1)N}\left(\sum_{i=1}^{N-1}\sum_{K=i+1}^{N}{\overset{ˆ}{\mathrm{Corr}}}_{i,t}\right)}$$

#### 3.3.3 Unit root test

The tests of unit root conducted by Pedroni (2001) and Kao and Chiang (2001) have the potential to provide erroneous findings due to SH and CSD (Dogan and Seker, 2016). For this reason, researchers decided to utilize a unit root test, which is a second-generation test devised by Pesaran (2007) and known as CIPS. The purpose of this test was to establish whether or not the variables involved in the CSD existence and slope heterogeneity were stationary. A cross-sectional average of $t_{i}$ is required to derive an estimator of CIPS, as established in the accompanying illustration in Equation (7):

(7) $$\mathrm{CIPS}=\frac{1}{N}\sum_{i=1}^{N}t_{i}(N,T)$$

On the other hand, Cross-sectional Augmented Dicky Fuller (CADF) test is highly related to the CIPS test. The CADF can be calculated as follows in Equation (8):

(8) $$\Delta Y_{it}=\varphi_{i}+\zeta_{i}Y_{i,t-1}+\delta_{i}{\underline{Y}}_{t-1}+\sum_{j=0}^{P}\delta_{ij}{\underline{Y}}_{t-1}+\sum_{j=1}^{P}\lambda_{ij}\Delta Y_{i,t-1}+\varepsilon_{it}$$

Where ${\underline{Y}}_{t-1}$ and $\Delta Y_{i,t-1}$ are the average for the lagged value and the first difference value of each cross-sectional series.

#### 3.3.4 Co-integration test

Since the first generation of co-integration tests (Rolf et al., 2001; Pedroni, 2004; Westerlund, 2005) do not take into account the influence of CSD, it is impossible to anticipate the features of panel data size distortion using those tests. However, even when analyzing data collected in a cross-sectional manner, Kao and Chiang (1998) and Pedroni (2001) failed to take CSD into account. Because of the CSD and the heterogeneity of the data, as well as the fact that the data are non-stationary, this approach is utilized to determine whether or not there is cointegration. The approach of data analysis that takes into account heterogeneity in slope, coefficient of variation, and correlated errors is one that was developed by Westerlund and Edgerton (2008). The second-generation panel co-integration technique (Westerlund, 2007) was applied in this analysis to visualize the co-integration linkages among the variables applied in this investigation. Using this method, it is possible to estimate properties of co-integration in the CSD of heterogeneous panel data sets with high confidence.

An overall description of four-panel cointegration tests is shown in the following Equations (9), (10), (11), and (12):

(9) $$G_{t}=\frac{1}{n}\sum_{i=1}^{N}\frac{T{\overset{´}{\alpha }}_{i}}{{\overset{´}{\alpha }}_{i}(1)}$$

(10) $$G_{a}=\frac{1}{n}\sum_{i=1}^{N}\frac{{\overset{´}{\alpha }}_{i}}{SE({\overset{´}{\alpha }}_{i})}$$

(11) $$P_{t}=\frac{\overset{´}{\alpha }}{SE(\overset{´}{\alpha })}$$

(12) $$P_{a}=T\overset{´}{\alpha }$$

In the aforementioned equations, $P_{t}$ and $P_{\alpha }$ are here panel cointegration and $G_{t}$ and $G_{\alpha }$ are the group mean statistics. The null hypothesis claims that the variables in the model do not have co-integrating linkages.

#### 3.3.5 CS-ARDL test

Following the Westerlund (2007) panel co-integration test, our study will employ the newest approach of CS-ARDL with several other related estimators like MG, AMG, and CCEMG. The well-known CS-ARDL test, designed by Chudik et al. (2016), can be utilized for both long-term and short-term evaluations here. When compared to other techniques like the MG, PMG, CCEMG, AMG, and GMM, this one is superior in terms of accuracy and reliability (Wang et al., 2021). Heterogeneity in slope, CSD, mixed-order integration in unit root tests, and the endogeneity problem are all issues that are made clearer by this method. The failure to account for common components not directly observed causes these issues and yields inaccurate estimation results. The succeeding Equation (13) represents the CS-ARDL model:

The model equation may be written as:

(13) $$L\mathrm{CO}2=\alpha_{it}+\sum_{j=1}^{P}\beta_{it}L\mathrm{CO}2_{i,t-j}+\sum_{j=0}^{P}\gamma_{it}X_{t-j}+\sum_{j=0}^{3}\delta {\underline{Y}}_{t-j}+\varepsilon_{it}$$

Where

$$\bar{Y_{t}}={\left(\Delta \bar{L\mathrm{CO}2_{t}},\bar{X_{t}}\;\prime \right)}^{\prime }\;\text{and}\;X_{it}={\left(L{\mathrm{GDP}}_{it}L{\mathrm{REN}}_{it}L{\mathrm{ENER}}_{it}L{\mathrm{NUC}}_{it}LR\&D\right)}^{\prime }.$$

## 4 Findings

The findings of homogeneity of the slope test advanced by Pesaran and Yamagata (2008) are presented in Table 3. It demonstrates that the model has a heterogeneity problem that has to be addressed. This suggests that the model contains coefficients that are not homogeneous, and that's why the slope of the line differs depending on the country. The rejection of homogeneity of slope means that the causality in panel analysis can lead to wrong conclusions if it imposes a restriction of homogeneity on the variable of interest.

**Table 3:** Slope homogeneity test.

SH tests	*Δ* statistic	P-value
$\overset{ˇ}{\Delta }$ test	12.615***	0.000
${\overset{ˇ}{\Delta }}_{\mathrm{adj}}$ test	16.960***	0.001

*A test for slope heterogeneity is predicated on the assumption that all slope coefficients are similar*. Asterisks (***) denote statistically significant values at the 1% level.

Before diving into an econometric study of panel data, it is essential to ensure CSD. As summarized by Pesaran's (2015) test, their results show signs of cross-sectional dependence. Because of the many shared economic, social, and political characteristics of the EU region, Table 4 shows a strong cross-sectional correlation between CO2, GDP, REN, ENER, R&D, and NUC. Given the scale of the EU economy in comparison to the rest of the globe, this is to be anticipated. In addition, these countries have similar policies regarding issues such as commerce, tourism, education, and employment.

**Table 4:** Result of CSD test.

Variable	Test Statistics (P-value)
*LCO2*	14.03***
*LGDP*	120.12***
LGDP^2^	140.05***
*LREN*	38.83***
*LENER*	15.14***
*LNUC*	20.00***
*LR&D*	11.96***

Note: Asterisks (***) denote statistically significant values at the 1% level.

Next-generation tests include panel unit root and co-integration, which follow the CSD test and the slope homogeneity test. Verifying the stationary test is next. For this reason, Table 5a, Table 5b detail the outcomes of the unit root test. An inherently asymmetric order of integration across all variables has been established. This means they are not following the same trend as other economic indicators like CO2, GDP, REN, ENER, R&D, and NUC. It is crucial to do a panel data analysis to verify the stationarity of a group of variables. The results of the 2nd generation unit root tests are presented in Table 5a, Table 5b, which demonstrate that certain variables are stationary at the label (I(0)), while others become stationary after the first difference (I(1)), but none of the variables are fixed second order or I(2).

**Table 5a:** CIPS unit root test.

Variables	Level		First difference		Order
	Without trend	With trend	Without trend	With trend	
*LCO2*	−1.902	−2.004	−3.642***	−3.784***	I(1)
*LGDP*	−1.250	−2.114	−3.218***	−3.846***	I(1)
*LGDP*_*2*_	−2.630***	−2.774***	−2.957***	−3.472***	I(0)
*LREN*	−3.014***	−3.254***	−4.541***	−4.840***	I(0)
*LENER*	−1.240	−1.356	−2.597***	−3.524***	I(1)
*LNUC*	−2.864***	−3.024***	−4.014***	−5.106***	I(0)
*LR&D*	−0.048	−1.854	−3.014***	−5.014***	I(1)

**Note:** The *, **, and *** denote the 10%, 5%, and 1% levels of significance, respectively.

**Table 5b:** CADF unit root test.

Variable	CADF test					
	At Level			1^st^ differences		
	T-bar	Z-t-tilde-bar	P value	T-bar	Z-t-tilde-bar	P value
*LCO2*	−2.485	−1.671	0.47			
*LGDP*	−2.606	−1.966	0.025			
*LGDP*^*2*^	−2.041	−0.621	0.267	−3.051	−3.023	0.001
*LREN*	−2.333	−1.320	0.093			
*LENER*	−1.173	1.444	0.926	−4.745	−7.053	0.000
*LNUC*	−1.015	−1.452	0.074			
*LRD*	−1.794	−0.034	0.486	−4.983	−7.620	0.000

Four of the variables in Table 5b are at level (I(0)) and three are at the first difference (I(1)). Contrarily, at the second difference or I(2), none of the variables are held constant.

After ensuring that all variables are indeed stationary, it is time to look into whether or not they are cointegrated across longer periods. Table 6 displays the results of the co-integration tests conducted in our study, which were developed using the work of Westerlund (2007). The p-values show that the null hypothesis given by Westerlund (2007) is not accepted at the various significance levels. The p-values for the Gt and Ga statistics are significant (less than 10%) and we can rule out the null hypothesis. Three of the four test statistics are statistically significant. Both group and panel cointegration tests provide similar findings, demonstrating the existence of a long-run cointegration connection between the variables studied in the EU region. AIC values are used to determine the maximum lag times. Our long-term variables are therefore co-integrated. According to the above discussion, it is narrated that variables co-integrate over a long period.

**Table 6:** Co-integration tests.

Statistic	Value	Z-value	P-value
*Gt*	−3.412	−1.174	0.010
*Ga*	−5.264	2.356	0.060
*Pt*	−4.404	2.254	0.450
*Pa*	−3.886	2.741	0.030

The CS-ARDL model can be shown in Table 7, and it is composed of both our long-term and short-term foundation models, respectively. Table 8 of the study includes applications of the MG, AMG, and CCEMG estimators, thus their robustness is examined. According to claims, *GDP* has a negative coefficient and has both short- and long-term effects on *CO2 emissions*; this implies that if *GDP* rises by 1%, *CO2 emissions* decrease by 0.779 percent and 1.720 percent, respectively. This result is similar to Amarante et al. (2021), Al-mulali et al. (2016), Ahmed (2020), Akif and Asumadu (2019), Prince and Okechukwu (2019), Liu et al. (2020), Voumik et al. (2022b) and Vo and Vo (2019) and the result is contradicted to Ozgur et al. (2022), Safi et al. (2021), Tao et al. (2021), Acaravci and Ozturk (2010), Ahmed et al. (2020), Aydin et al. (2019), Awais and Wang (2019), Abbasi et al. (2020), Bano et al. (2018), Tauseef et al. (2019), Erdogan et al. (2020), Fakher (2019), Marrero (2010), and Liu et al. (2020). By contrast, the coefficient of ${\mathrm{GDP}}^{2}$ is positive and significant statistically, which shows that if ${\mathrm{GDP}}^{2}$ rises by 1 percent, then it increases ${\mathrm{CO}}_{2}$ emissions by 0.0124 percent. This result is produced by Aydin et al. (2019), Awais and Wang (2019), Akif and Asumadu (2019), Dogan et al. (2020), Marrero (2010), and contradicts Ozgur et al. (2022), Tao et al. (2021), Acaravci and Ozturk (2010), Ahmed et al. (2020), Akif and Asumadu (2019), Erdogan et al. (2020), Dogan et al. (2020), and Vo and Vo (2019). Renewable energy reduces CO2 emissions; that is, if renewable energy consumption increases by 1%, CO2 emissions are reduced by .1129 percent. This result is similar to Haldar and Sethi (2021), Esquivias et al. (2022), Sahoo and Sethi (2021), Amarante et al. (2021), Al-mulali et al. (2016), Erdogan et al. (2020), Marrero (2010), Prince and Okechukwu (2019), Liu et al. (2020), and Voumik et al. (2022c). Furthermore, the energy intensity coefficient value is .3953, which is both positive and significant, indicating that if energy intensity increases by 1%, CO2 emissions increase by .3953%. This is similar to Sethi and Dash (2022), Ahmed (2020), Abbasi et al. (2020), Bano et al. (2018), Akif and Asumadu (2019), Fakher (2019), and Marrero (2010). The impacts of nuclear energy on *CO2 emissions* in the long-term context are negative but insignificant, and similar results are produced by Ozgur et al. (2022) and Bezi (2022). And the coefficient of research and development is −.9114, which is also negative and ensures its statistical significance. That means research and development minimize *CO2 emissions*, and if the research and development budget is increased by 1%, then the *CO2 emissions* decrease by .9114%. The same outcome is produced by Safi et al. (2021) and Tao et al. (2021).

**Table 7:** CS-ARDL test.

Variables	Long-run coefficients	Short-run coefficients
*LGDP*	−0.779**(7.7686)	−1.720***(6.486)
*LGDP*^*2*^	0.0124*(0.5969)	0.03113*(4.1324)
*LREN*	−0.1129***(0.5905)	−0.035(0.4440)
*LENER*	0.3953**(0.2734)	0.2785**(0.2074)
*LNUC*	−0.142(0.196)	−0.0117(0.0231)
*LRD*	−0.024**(0.024)	−0.0112***(0.0146)
**Adjusted Term**	−0.7114***(0.1150)	
Number of groups	34	
R-squared	0.444	

Error estimates within brackets.

*** p<0.01, ** p<0.05, * p<0.1.

**Table 8:** Robustness check.

Variables	AMG	MG	CCEMG
LGDP	−1.609(8.936)	−1.250(6.722)	−0.260(5.299)
LGDP^2^	0.0422**(0.171)	0.0196(0.131)	0.0355*(0.112)
LREN	−0.169***(0.0456)	−0.182***(0.0492)	−0.131**(0.0556)
LENER	0.885***(0.0736)	0.941***(0.0652)	0.936***(0.0816)
LNUC	−0.0432**(0.0368)	−0.0386*(0.0367)	−0.0488(0.0338)
LRD	−0.0311(0.0262)	−0.0255(0.0207)	−0.0378*(0.0416)
Constant	7.765(117.0)	23.80(86.42)	9.976(72.80)
Observations	571	571	571
Number of ids	31	31	31

Error estimates within brackets.

*** p<0.01, ** p<0.05, * p<0.1.

Short-term statistical significance exists for the *GDP* coefficient, which is negative and represents a 1% rise in *GDP*, which would reduce *CO2* emissions by 1.720. The same output is produced by Ahmed et al. (2020) and Tauseef et al. (2019), and *GDP2*'s slope coefficient is positive and significant, and the same output is consistent with Ahmed et al. (2020). Renewable energy's short-run coefficient value indicates that it minimizes CO_2_ but insignificant. The energy intensity coefficient is significant and positive in this instance, which indicates that if energy intensity increases by 1%, then ${\mathrm{CO}}_{2}$ *emissions* increase by .2785%. The same findings are concluded by Bano et al. (2018). The nuclear energy coefficient is −.0117, which means that every 1% increase in nuclear energy consumption reduces greenhouse gas emissions by .0117%. The research and development coefficient value are −.0112, which is negative and also significant, which shows that if *research and development* sector improvements increase by 1%, then *CO2* emissions reduce by .0112%. Overall, the goodness of fit (R^2^) is 0.344, which states that only 34% of the variation in ${\mathrm{CO}}_{2}$ emissions is explained by *GDP*, ${\mathrm{GDP}}^{2}$, *renewable energy*, *energy consumption*, and *R&D*.

Table 8 explains the robustness results, and to observe robustness among the variables, the methods of CCEMG, AMG, and MG were applied. The EKC hypothesis also exists in these three methods, though most of the coefficients are insignificant. The coefficients of renewable energy are negative and significant for all estimators. Similarly, the coefficients for nuclear energy are also negative and significant for the AMG and MG estimators. Research and development coefficients are negative, but all are insignificant. On the other hand, coefficients for energy intensity are detrimental to the environment, and all coefficients are highly significant.

## 5 Discussion

The concluding results of Table 7 demonstrate that *GDP* promotes environmental standards. This is because of the application of new green technology in industry or production houses; therefore, a greater proportion of production emits fewer emissions and ensures ecological sustainability. When a larger number of renewable energies are used in production and the heat released in the atmosphere is carbon-free, consequently, economic growth occurs but pollution concerning the environment decreases. Amarante et al. (2021), Ahmed (2020), Dogan et al. (2020), and Liu et al. (2020) also found the same results: *GDP* enhances environmental compatibility. By contrast, the *GDP square* is responsible for environmental degradation, which means in the production process, a greater number of non-renewable energies or backdated technologies are used, which emit more emissions, and consequently, an increase in production generates a higher level of pollution. Some researchers, including Dogan et al. (2020), Marrero (2010), and Vo and Vo (2019), claim that GDP2 has a negative impact on the environment. *Renewable energy* fuels are carbon-free. It emits fewer emissions than other energy sources but produces more energy than is used in production. *Renewable energy is energy that comes from sources that are all around us, such as the sun, water, waste, and wind, and is replenished by nature with heat from the earth. These sources do not emit harmful carbon dioxide, and thus emit little or no pollutants into the air*. Thus, it has a detrimental effect on the pollution of the environment Earlier researchers, for instance, Haldar and Sethi (2021) and Esquivias et al. (2022), also found the same outcomes in their research. Again, by contrast, by burning non-renewable energy like oil and coal, large amounts of nitrogen oxides enter the air and result in acid rain and smog, which means producing and burning fossil fuels creates a favorable environmental effect and produces greenhouse gas emissions. Thus, energy intensity has an unfavorable impact on the environment. *Nuclear energy* is known as a zero-emission, clean energy source that maintains air quality. *Nuclear energy* is produced by the process of fission, which produces energy by splitting uranium atoms. It produces electricity by spinning turbines, without any harmful byproducts. As a result, nuclear energy negatively impacts greenhouse gas emissions. Recent research conducted by Ozgur et al. (2022) and Bezi (2022) also indicated that nuclear energy is really good for maintaining the quality level of the environment. It is also observed that research and development have a detrimental impact, as more *R&D* means better environmental quality and less ${\mathrm{CO}}_{2}$. This is because by doing *RD*, more environmentally friendly energy is discovered, and people are becoming concerned about it and finding alternative sources of non-renewable power; thus, *R&D* improves environmental compatibility.

## 6 Conclusion

The major objective of this analysis is to evaluate how *GDP*, ${\mathrm{GDP}}^{2}$, *renewable energy*, *nuclear energy*, and *research and development* are accountable for determining environmental quality, using panel data analysis for the European Union countries from 1991 to 2021. The variables' stationarity is tested using the CIPS and CADF, which are second-generation unit root tests, and the long-run equilibrium is studied using a panel co-integration (Westerlund, 2007) analysis of the second-generation test. Cross-sectional methods are used to determine whether or not the variables are interdependent. To assess the stability of the associations between variables over time, this study employed a cutting-edge technique known as the CS-ARDL. Our long-run variables are co-integrated, as shown by Westerlund's panel co-integration test. The results of CS-ARDL show that *GDP*, *renewable energy*, *nuclear energy*, and *RD* can minimize ${\mathrm{CO}}_{2}$ *emissions*, while ${\mathrm{GDP}}_{2}$ and *energy intensity* increase ${\mathrm{CO}}_{2}$ *emissions* in the European Union. And, *GDP, renewable energy, and RD* are statistically significant in the long term to lessen environmental deterioration levels. The EKC hypothesis is not supported by these findings, which show that as economic growth rises, so does environmental pollution and that ${\mathrm{CO}}_{2}$ levels eventually rise. In the EKC hypothesis, after a certain point of economic growth, environmental degradation slows down and reflects a systematic and deterministic linkage, as demonstrated by the EKC, according to Grossman and Krueger (1991). In addition to confirming a long-lasting relationship within the variables, AMG, MG, and CCEMG tests are applied, and these tests indicate that *GDP, renewable energy, nuclear energy, and research and development* can assure environmental compatibility because these indicators help reduce environmental deterioration. So, the robustness test provides additional evidence that the methodology and the CS-ARDL technique are suitable for the task at hand. This study also recommends increasing production by applying cleaner and greener energy in places where usage of non-renewable energy raises greenhouse gas emissions, such as increasing renewable energy, and nuclear energy use, and investing more in the research and development sector.

## 7 Policy recommendation

The European Union is facing continuous threats from its major energy supplier, the Russian Federation. Because most of the nonrenewable energy that EU countries use comes from Russia, which is a clear threat to these countries, they are trying to use less nonrenewable energy. Our research supports their ongoing energy-saving activities in a different sector. Based on the findings and conclusion, several policies must be set for the European Union.

• From our findings, it is known that *GDP* reduces greenhouse gas emissions, so the policymakers of the EU should focus on the production sector because more production is significantly reducing greenhouse gas emissions, which means more economic growth leads to less environmental deterioration. Definitely, in the production process, green technology-based equipment should be implemented so that production will increase and, at the same time, environmental sustainability will also be ensured. Moreover, the policymakers can also take another step to provide subsidies, monthly allowances, or yearly bonuses to those firms that use green technology, and they should follow strict rules to ban such kinds of production equipment that produce more emissions.
• Although *GDP* improves environmental quality, ${\mathrm{GDP}}^{2}$ leads to environmental degradation. This may have happened by using high-emitting technologies, which are cheap but create a serious threat to our environment. So, the policymakers of the European Union should create a straight law so that every industry or firm is compelled to follow the rules of using green technology and should have a system of punishment if anyone breaks the rules. Only after this will environmental compatibility be possible; otherwise, it will not be.
• As *renewable energy* negatively and statistically impacts greenhouse gas emissions, EU policymakers can implement greenery and clean equipment, and as a result, *renewable energy* will increase, energy scrutiny will improve, and the dependability of energy on non-renewable sources will decline. In addition, when the consumption of non-renewable energy declines, it plays a crucial role in mitigating ${\mathrm{CO}}_{2}$ *emissions*. Furthermore, governments should find new sources of renewable energy so that no one has to rely on non-renewable energy. Besides, governments can also raise the price of non-renewable energy so that the demand for it declines.
• *Energy intensity* increases environmental pollution, so policymakers should encourage people to switch energy consumption and move to *renewable energy sources* such as tidal energy, breeze energy, hydroelectricity, biomass energy, and geothermal energy, as the consumption of *non-renewable energy* is alarming in the European Union. As we know, these renewable sources don't have any devastating impacts on the environment, and they are friendly to a green environment. Also, governments can set up different programs to make people more aware of the environment and the bad things that happen when people use too much energy.
• It is also seen that nuclear energy minimizes ${\mathrm{CO}}_{2}$ *emissions*. So, the government should build more nuclear energy plants so that the reliability of non-renewable resources can be avoided. There is an urgent need to increase investment in research, innovation, and development projects in European Union countries. Additionally, the government can provide various incentives to the people so that they are encouraged to use nuclear energy to maintain environmental compatibility.
• *R&D* sectors help to alleviate greenhouse gas emissions. In this case, the government must cooperate in the research sector and with innovative technology so that researchers and scientists can find alternative sources of green energy to fulfill present and future energy demands. It is also known that non-renewable resources are scarce, so it is a wise decision for the EU to depend on renewable resources to have time. The quality regulation authorities should establish rules and regulations for renewable energy, observe the activities, and try to achieve sustainable development. They should arrange programs to raise awareness about the negative impact of *CO2 emissions* and encourage them to use renewable resources instead of non-renewable resources.

## 8 Future research and limitations

While this study has its limitations, they may point to important avenues for further study. Firstly, this study does not cover the world's largest CO_2_ emitters, like China, the USA, India, Brazil, South Africa, and other countries that are responsible for emitting most of the carbon dioxide in the world. Secondly, this study did not consider variables like green finance, institutional quality, etc. as the key variables of the environment-related study. Further research may contain these variables as independent variables to explain the EKC hypothesis. Thirdly, this study did not consider the overall economic impact of COVID-19, various shocks, or structural breaks. Future research may adjust these impacts to explain the EKC hypothesis with renewable energy consumption, nuclear energy, and R&D for the EU. The data of this research is imbalanced panel data, and there are a lot of missing observations. Future research will overcome this. The research applied the CS-ARDL method; future research will apply more updated econometric tools.

## Declarations

### Author contribution statement

Liton Chandra Voumik: Conceived and designed the experiments Contributed reagents, materials, analysis tools, or data; Wrote the paper.

Mahbubur Rahman: Performed the experiments; Analyzed and interpreted the data.

Salma Akter: Performed the experiments; Wrote the paper.

### Funding statement

This research did not receive any specific grant from funding agencies in the public, commercial, or not-for-profit sectors.

### Data availability statement

Data will be made available on request.

### Declaration of interests statement

The authors declare no competing interests.

### Additional information

No additional information is available for this paper.
